This article has been retracted.

# Polymyxin B, Cefoperazone Sodium-Sulbactam Sodium, and Tigecycline against Multidrug-Resistant *Acinetobacter baumannii* Pneumonia

**DOI:** 10.1155/2022/1968020

**Published:** 2022-05-31

**Authors:** Guangxue Hu, Wanzong Liu, Mali Wang

**Affiliations:** Laboratory Department, The Fifth People's Hospital of Wuhu, Wuhu, Anhui Province, China

## Abstract

**Purpose:**

The purpose of this study is to investigate the significance of polymyxin B in combination with cefoperazone sodium-sulbactam sodium (CSSS) and tigecycline for the treatment of multidrug-resistant *Acinetobacter baumannii*- (MDRAB-) induced pneumonia on the levels of white blood cell (WBC) count, serum C-reactive protein (CRP), and procalcitonin (PCT).

**Methods:**

Fifty-six patients with MDRAB pneumonia admitted to the Fifth People's Hospital of Wuhu from February 2019 to December 2021 were randomized into the observation group (*n* = 28) and the experimental group (*n* = 28) by the random table method. The observation group received intravenous infusion of CSSS and tigecycline. The experimental group received intravenous infusion of polymyxin B sulfate plus CSSS and tigecycline. All patients were treated for 14 days.

**Results:**

There was no significant difference in the overall response rate between the two groups; the bacterial clearance of the experimental group was significantly higher than that of the observation group; there was no significant difference in the WBC, CRP, and PCT levels between the two groups prior to the treatment; but after treatment, while the WBC, CRP, and PCT levels of the two groups decreased, the WBC count, CRP, and PCT levels of the experimental group were significantly lower than those of the observation group; no significant difference was found in adverse reactions.

**Conclusion:**

Polymyxin B-CSSS-tigecycline has good clinical efficacy in the treatment of MDRAB pneumonia. It not only improves the patients' bacterial clearance rate and effectively reduces the levels of WBC count, serum CRP, and PCT, but also raises no risk of adverse reactions. Therefore, it is worthy of clinical promotion.

## 1. Introduction

*Acinetobacter baumannii* (*A. baumannii*) is a nonfermenting Gram-negative bacterium, which exists widely in nature. It is an opportunistic pathogen with a strong ability to replicate and clone, and its rapid transmission brings about its worldwide prevalence [1, 2]. *A. baumannii* is clinically common and possesses strong environmental adaptability and long survival period [3]. Multidrug-resistant *A. baumannii* (MDRAB) is one of the main causes of hospital-acquired infections and critical patient deaths [4]. It can trigger enormous danger by inducing respiratory infections, bacteremia, surgical site infections, infectious meningitis, infectious pneumonia, and other diseases, and its disability rate and mortality rate rank top among all types of bacterial infections [5]. *A. baumannii* has a variety of drug resistance mechanisms, including beta-lactamase, efferent pump activation and overexpression, membrane permeability reduction, change of penicillin binding protein, and enzymatic modification of aminoglycosides. The main mechanism of drug resistance to hydrocarbapenes is hydrocarbapenase production [6].

According to prior studies, a combination of multiple antimicrobial drugs and antimicrobial synergists is needed given that the single drug against MDRAB works unsatisfactorily [7]. In treating pneumonia induced by MDRAB, cefoperazone sodium-sulbactam sodium (CSSS) and tigecycline are often used, yet as the time prolongs, resistance of MDRAB increases leading to weakening efficacy of the medicine [8]; polymyxin B is an antibiotic that shows great effectiveness in treating many pathogenic diseases [9]. The white blood cell (WBC) count and serum C-reactive protein (CPR) are both common infectious disease detection indicators, but some studies have demonstrated their unsatisfactory detection effect [10], so further clinical analysis is still in need; procalcitonin (PCT) is a common precursor of calcitonin in laboratory tests, and its level increases distinctively in MDRAB pneumonia, as explained in relevant medical studies [11]. In this study, 56 patients with MDRAB pneumonia admitted to our hospital from February 2019 to December 2021 were selected to explore the significance of polymyxin B-CSSS-tigecycline for the treatment of the disease on the levels of WBC count, serum CRP, and PCT, so as to provide clinical reference.

## 2. Materials and Methods

### 2.1. General Profile

Fifty-six patients with MDRAB pneumonia admitted to the Fifth People's Hospital of Wuhu from February 2019 to December 2021 were randomized into 2 groups, the observation group (*n* = 28) and the experimental group (*n* = 28), by the random table method. All patients and families were informed of the study and signed the consent form. The study protocol was approved by the Ethics Committee of the Fifth People's Hospital of Wuhu in accordance with the ethical guidelines for clinical research (approval no. 2018-LS231).

### 2.2. Inclusion and Exclusion Criteria

#### 2.2.1. Inclusion Criteria

The inclusion criteria were as follows: age >18 years, meet the diagnostic criteria for hospital-acquired pneumonia (HAP), *A. baumannii* was isolated from selected sputum and alveolar lavage fluid for two consecutive times, and pathogenic bacteria isolated from the sputum was ≥10^6 cfu/mL.

#### 2.2.2. Exclusion Criteria

The exclusion criteria were as follows: patients with cardiac, hepatic, renal insufficiency, or other serious infections; immune diseases and malignant tumors; mental disorders; allergy to therapeutic drugs; and pregnancy or lactating mother.

### 2.3. Methods

All patients were treated with sputum cultures and symptomatic medication after admission. Those in the observation group were given intravenous infusion of CSSS (Pfizer Pharmaceutical Co., Ltd., approval number H20020598, specification: 1.5 g/stick, batch number: AM3387, AM3648) every 12 hours with 3 g added to 0.9% sodium chloride solution, and 2 hours later, they were given intravenous infusion of tigecycline (Jiangsu Hansoh Pharma, approval number H20123394, specification: 50 mg/stick, batch number: 81711011, 81803031), 100 mg at first dose, and then 50 mg every 12 hours for maintenance, 2 times/day. Other than the same treatment as in the observation group, patients in the experimental group were given intravenous infusion of polymyxin B sulfate (SPH First Biochemical and Pharmaceutical Co., Ltd., SFDA approval number: H31022631, specification: 500,000 units, batch number: 2002803, 2006801), 1–1.5 million units/day at 2-3 intervals. Both groups of patients were treated for 14 days.

### 2.4. Observation Indicators and Evaluation Criteria

#### 2.4.1. Clinical Efficacy

Clinical efficacy was evaluated after 14 days of treatment in accordance with the consensus of MDR bacteria control experts and was categorized into excellent (patients' clinical signs and symptoms as well as all indicators showed significant improvement), effective (patients' clinical signs and symptoms as well as all indicators showed certain improvement), and ineffective (patients' clinical signs and symptoms did not improve or even worsened). Overall response rate = (excellent + effective) × number of cases/total number of cases × 100%.

#### 2.4.2. Peripheral Blood Test Indexes

Serum indicators included WBC count, serum CRP, and PCT. Prior to and after treatment, 5 ml each of fasting venous blood was drawn from the patients in the early morning, and serum was isolated after high-speed centrifugation and standing. Serum PCT was detected using a PCT test kit (Guangzhou Wanfu Biotechnology Co., Ltd.). CRP detection was performed by a CRP detection kit (Zhejiang Meikang Biological Co., Ltd.), and the WBC count was detected by an XN-1000 automatic blood cell analyzer (Japan SYSMEX Co., Ltd.).

#### 2.4.3. Bacterial Clearance Rate

After antibacterial drug discontinuation, multiple qualified specimens were taken and sent for bacteria culture to evaluate bacterial clearance, which was categorized into cleared (qualified posttreatment specimen was taken and sent for bacteria culture and the results suggested no growth of pathogenic bacteria), assumed cleared (patients' posttreatment clinical signs of infection significantly improved, but the qualified bacteria were unable to be collected), replaced (original pathogenic bacteria within the patients were eradicated after treatment, but new ones were suggested from the bacterial culture results though no clinical symptoms were presented), and uncleared (posttreatment pathogenic bacteria still existed). Bacterial clearance rate = (clearance + assumed clearance) × number of cases/total number of isolates.

#### 2.4.4. Adverse Reactions

Adverse reactions during the treatment were observed and recorded, including nausea and vomiting, chest tightness and shortness of breath, and gastrointestinal discomfort.

### 2.5. Statistical Methods

SPSS 21.0 software was used for data analysis, measurement data were expressed as ($\bar{x}$±*s*), and independent sample *t*-tests were used; enumeration data were presented as (*n*, %), and the chi-square test was used. *P* < 0.05 indicated statistical significance.

## 3. Results

### 3.1. General Profile

The observation group consisted of 19 males and 9 females, aged (71.64 ± 12.38) years, with the APACHE-II scores of (26.41 ± 1.57) points and GCS scores of (11.55 ± 1.68) points. The experimental group consisted of 21 males and 7 females, aged (69.36 ± 17.90) years, with the APACHE-II scores of (26.35 ± 1.61) points and GCS scores of (11.70 ± 1.59) points. The differences in gender, age, APACHE-II score, and GCS score between the two groups were statistically nonsignificant (*P* < 0.05) (Table 1).

### 3.2. Comparison of Clinical Efficacy

In the observation group, there were 8 cases of excellent efficacy, 14 cases of effective efficacy, and 6 cases of ineffective efficacy, with an overall response rate of 78.57% (22/28). In the experimental group, there were 11 cases of excellent efficacy, 12 cases of effective efficacy, and 5 cases of ineffective efficacy, with an overall response rate of 82.14% (23/28). No significant difference was found between the two groups in the overall response rate (*P* > 0.05) (Table 2).

### 3.3. Comparison of Bacterial Clearance Rate

In the observation group, there were 8 cases of the cleared, 5 cases of the assumed cleared, 9 cases of the replaced, and 6 cases of the uncleared, with a clearance rate of 46.63% (13/28). In the experimental group, there were 12 cases of the cleared, 9 cases of the assumed cleared, 4 cases of the replaced, and 3 cases of the uncleared, with a clearance rate of 75.00% (21/28). The bacterial clearance rate of patients in the experimental group was significantly higher than in the observation group (*P* < 0.05) (Table 3).

### 3.4. Comparison of Serum Indicators

No significant differences were shown in the WBC, CRP, and PCT levels between the two groups prior to the treatment (*P* < 0.05); after treatment, the WBC, CRP, and PCT levels of the two groups decreased (*P* < 0.05), and the WBC, CRP, and PCT levels of patients in the experimental group were significantly lower than those in the observation group (*P* < 0.05) (Table 4).

### 3.5. Comparison of Adverse Reactions

In the observation group, there was 1 case of nausea and vomiting, 1 case of chest tightness and breath shortness, and 1 case of gastrointestinal discomfort, with an overall rate of 10.71% (3/28). In the experimental group, there were 2 cases of nausea and vomiting, 1 case of chest tightness and breath shortness, and 1 case of gastrointestinal discomfort, with an overall rate of 14.29% (4/28). No significant difference in the patients' adverse reactions was seen between the two groups (*P* < 0.05) (Table 5).

## 4. Discussion

*A. baumannii* is widely distributed, especially at hospital where the patient's immunity is affected and antibiotics and other invasive devices are clinically used, significantly raising the patient's infection rate [12]. This highly resistant bacterium possesses resistance mechanisms against many antibiotics, such as active efflux pump systems and accumulation of integron-mediated resistance genes [13]. Now, MDRAB pneumonia has become one of the main health-threatening diseases, and if not treated in time, patients will face damages in the heart, liver, kidney, and other important organs, which will trigger more complications and hamper prognosis [14]. Drug therapy is the major treatment regimen against MDRAB pneumonia, and clinically effective drugs include *β*-lactam and *β*-lactamase inhibitor combination, 3rd or 4th generation cephalosporins, fluoroquinolones, and aminoglycosides. A combined use of these drugs is recommended by numerous clinical studies [15]. It has been confirmed by clinical studies that cefoperazone-sulbactam can effectively inhibit *β*-lactamase and quickly kill *Acinetobacter*, while tigecycline is another drug against *A. baumannii* that can invalidate the bacterial protein synthesis, and a combination of these two can remarkably reduce the occurrence of *A. baumannii* resistance. Polymyxin B was once clinically banned mainly for its high nephrotoxicity and neurotoxicity, yet as antibiotic resistance keeps growing; polymyxin B is readopted in the medical treatment against infection by the drug-resistant *A. baumannii* and for preventing disease resistance, forming a hot research focus [16]. The national bacterial resistance surveillance showed that polymyxin B has a sensitivity rate of over 96% to *A. baumannii*. It also showed good in vitro antibacterial activity against *A. baumannii* when combined with rifampicin, carbapenems, tigecycline, aminoglycosides, ampicillin/sulbactam, and minocycline (two or three drugs combined) [17]. A randomized controlled clinical (RCT) study by Zhang Pingxing indicated that polymyxin B combined with rifampicin against MDRAB infection resulted in better bacterial clearance, even though no difference in mortality was found. In our study, we compared the clinical efficacy and bacterial clearance of two groups, and the results showed that there was no significant difference in the overall response rate between the two, but the bacterial clearance rate of the experimental group was significantly higher than that of the observation group, illustrating that whether CSSS or tigecycline combined with polymyxin B had no effect against MDRAB pneumonia, but polymyxin B-CSSS-tigecycline could notably improve the bacterial clearance rate. WBC count and serum CPR are both commonly used indicators to detect infection, but their detection effect is not ideal as explained in some studies, and thus, more clinical analyses are required. PCT is a more common precursor of calcitonin in laboratory tests, whose content, as shown in studies, increases significantly in MDRAB pneumonia [18]. We compared in this study the WBC, CRP, and PCT levels of the two groups and significant results were obtained. Prior to the treatment, there was no significant difference in the WBC, CRP, and PCT levels between the two groups; however, after treatment, the WBC, CRP, and PCT levels of both groups decreased, and the WBC, CRP, and PCT levels of the experimental group were significantly lower than those of the observation group, suggesting that polymyxin B-CSSS-tigecycline can effectively change the patient's WBC, CRP, and PCT levels, which is possibly because tigecycline as a new type of glycylcycline antibacterial drug can effectively inhibit the synthesis of bacterial proteins, prevent the aminoacylated tRNA molecules from entering the ribosomal A position by binding to the 30s ribosome subunit, and finally inhibit the synthesis of bacterial proteins and hinder the peptide chain extension when integrating the amino acid residue [19, 20]. Occurrence of adverse reactions during the treatment were compared to demonstrate medication safety, and the results showed that there was no significant difference between the two groups in this regard, proving that polymyxin B-CSSS-tigecycline syngenesis did not increase the risk of adverse reactions occurrence. However, this result is based on the small sample size of this study, and more clinical studies need to be conducted to confirm it [21].

Antibiotics play an irreplaceable role in the treatment of bacterial infectious diseases. However, due to the serious bacterial drug resistance, antibiotics appear “helpless” to solve the problem of bacterial drug resistance, so it is extremely urgent to find a new effective way to treat bacterial infectious diseases [22]. Chinese traditional medicine (TCM) is rich in resources with complex active components, hence possessing a wide antibacterial spectrum to act on multiple mechanisms of bacteria and play an antibacterial role. Therefore, TCM has become the focus of research on bacterial drug resistance. It has been demonstrated in a large number of literature that TCM has an inhibitory effect on the resistance of *A. baumannii*, and the combination of antibacterial TCM and antibiotics has a synergistic effect on the resistance of *A. baumannii*, providing a potential solution for bacterial resistance in the future [23].

However, this study has its own limitations as it was a single-center study with a small number of cases, a small sample size, and the patients in the study were characterized by relatively severe conditions, more medical procedures, and longer hospital stay, which inevitably resulted in result bias.

## 5. Conclusion

In conclusion, syngenetic use of polymyxin B-CSSS-tigecycline against MDRAB pneumonia could achieve good clinical efficacy. It not only could elevate the patient's bacterial clearance rate and effectively reduce the levels of WBC count, CRP, and PCT but also raise no risk of adverse reactions, and hence, it is worthwhile to be promoted clinically.

## Figures and Tables

**Table 1:** Comparison of general profile in the two groups.

	Observation group (*n* = 28)	Experimental group (*n* = 28)	*t*/*χ*^2^	*P*
Gender (male/female)	19/9	21/7	0.350	0.554
Age (years)	71.64 ± 12.38	69.36 ± 17.90	−0.500	0.621
APACHE-II score	26.41 ± 1.57	26.35 ± 1.61	0.719	0.858
GCS score	11.55 ± 1.68	11.70 ± 1.59	−0.435	0.665

APACHE, Acute Physiology and Chronic Health Evaluation; GCS, Glasgow Coma Scale.

**Table 2:** Comparison of clinical efficacy (*n*, %).

	Excellent	Effective	Ineffective	Response rate
Observation group (*n* = 28)	8	14	6	22 (78.57%)
Experimental group (*n* = 28)	11	12	5	23 (82.14%)
*χ* ^2^				0.113
*P*				0.737

**Table 3:** Comparison of bacterial clearance rate (*n*, %).

	Cleared	Assumed cleared	Replaced	Uncleared	Clearance rate
Observation group (*n* = 28)	8	5	9	6	13 (46.63%)
Experimental group (*n* = 28)	12	9	4	3	21 (75.00%)
*χ* ^2^					
*P*					

**Table 4:** Comparison of serum levels ($\bar{x}$ ± *s*).

Groups	WBC (×109/L)		CRP (mg/L)		PCT (mg/ml)	
	Before	After	Before	After	Before	After
Observation group (*n* = 28)	18.79 ± 4.71	11.38 ± 2.32	60.57 ± 20.12	44.32 ± 4.34	7.27 ± 1.21	2.35 ± 1.17
Experimental group (*n* = 28)	18.68 ± 4.65	9.12 ± 2.61	60.39 ± 20.14	30.58 ± 3.52	7.31 ± 1.15	1.71 ± 1.44
*t*	0.111	4.341	0.042	16.494	0.161	2.314
*P*	0.912	<0.001	0.967	<0.001	0.872	0.023

**Table 5:** Comparison of adverse reactions (*n*, %).

	Nausea and vomiting	Chest tightness and breath shortness	Gastrointestinal discomfort	Overall rate
Observation group (*n* = 28)	1	1	1	3 (10.71%)
Experimental group (*n* = 28)	2	1	1	4 (14.29%)
*χ* ^2^				0.163
*P*				0.686

## Data Availability

The data generated or analysed during this study are included within the article.
